# Assessing the Effects of Estrogen on the Dynamics of Breast Cancer

**DOI:** 10.1155/2012/473572

**Published:** 2012-12-19

**Authors:** Chipo Mufudza, Walter Sorofa, Edward T. Chiyaka

**Affiliations:** Modelling Biomedical Systems Research Group, Department of Applied Mathematics, National University of Science and Technology, P.O. Box AC 939, Ascot, Bulawayo, Zimbabwe

## Abstract

Worldwide, breast cancer has become the second most common cancer in women. The disease has currently been named the most deadly cancer in women but little is known on what causes the disease. We present the effects of estrogen as a risk factor on the dynamics of breast cancer. We develop a deterministic mathematical model showing general dynamics of breast cancer with immune response. This is a four-population model that includes tumor cells, host cells, immune cells, and estrogen. The effects of estrogen are then incorporated in the model. The results show that the presence of extra estrogen increases the risk of developing breast cancer.

## 1. Introduction

 Among many cancer types, breast cancer is the second most common cancer in women, exceeded only by skin cancers. The chance of developing invasive breast cancer at some time in a woman's life is a little less than about 12% [1]. Being exceeded only by lung cancer, breast cancer is the second leading cause of cancer deaths in women. The chance that breast cancer will be responsible for a woman's death is about 1 in 36 [1]. The disease has been more pronounced in the developed world in the past but has soon crossed boundaries into the developing world of Africa and Asia. In Zimbabwe, breast cancer is currently the third leading cancer responsible for deaths of women of all ages with crude mortality rate of 5.6 per 100 000, exceeded only by Cervical cancer and Kaposi sarcoma [2]. Breast cancer is a malignant (cancerous) tumor that starts in the cells of the breast, that is, a group of cancer cells that can grow into (invade) surrounding tissues or spread (metastasize) to distant areas of the body. It begins when breast cells start to grow out of control due to DNA damage which controls all cell actions in the body tissues. When DNA is damaged, normal cells will repair the damage or the cell dies but in cancer cells, damaged DNA is not repaired and does not die like it should. Instead the cell goes on making new abnormal cells with the same damaged DNA which the body does not need. A single genetically altered cell then grows into a tumor in a stepwise progression.

There are several types of breast cancer, but some of them are quite rare. In some cases a single breast tumor can be a combination of these types or be a mixture of invasive and *in situ* cancer. Ductal carcinoma *in situ* (DCIS) is the most common type of noninvasive breast cancer. DCIS means that the cancer cells are inside the ducts but have not spread through the walls of the ducts into the surrounding breast tissue. However, after starting in a milk passage (duct) of the breast, it can break through the wall of the duct and grow into the fatty tissue of the breast. At this point, it may be able to spread (metastasize) to other parts of the body through the lymphatic system and bloodstream and will now be referred to as invasive ductal carcinoma (IDC). Lobular carcinoma *in situ* (LCIS) is another type of noninvasive breast cancer which begins in the milk-producing glands and does not grow through the wall of the lobules. This can become invasive and spread to other parts of the body as invasive lobular carcinoma (ILC), a state which is harder to detect by a mammogram. 

## 2. Risk Factors and Vulnerable Groups

 There are many factors that affect the chance of an individual developing breast cancer, some of which one can change and some cannot be changed. Having a risk factor, or even several, does not mean that one will automatically develop the disease. Women have a higher risk of developing breast cancer although in men it has been discovered too [3]. Some of these factors include use of alcohol with the risk increasing relative to the amount of alcohol consumed, overweight or obese, especially for women after menopause. Obesity increases estrogen levels due to fat tissue producing small amounts of estrogen [1]. High doses of radiation are also known to increase breast cancer risk, where exposure to radiation from the atomic bomb at Hiroshima caused increased breast cancer incidence, especially in women exposed as teenagers, when their breast cells were very immature [4]. Repeated X-ray exposure for treatment of tuberculosis, postpartum mastitis, chest acne, and monitoring treatment for scoliosis increases risk [5]. A woman may become pregnant after a cancer cell has formed in her breast, a cell which may have been dormant for many years. However, with pregnancy, estrogen levels rise stimulating the dormant cancer cell to grow into a clinically detectable cancer [6].

Breast cancer incidence rates are higher in non-Hispanic white women compared to African American women for most age groups. Incidence and death rates for breast cancer are lower among women of other racial and ethnic groups like Asian, African, and Hispanic white than among non-Hispanic white and African American women [1]. However, in women under 45 years of age, breast cancer is more common in African American women. There is higher risk among women whose close blood relatives have this disease. Having one first-degree relative (mother, sister, or daughter) with breast cancer approximately doubles a woman's risk. Having 2 first-degree relatives increases her risk about 3-fold. The exact risk is not known, but women with a family history of breast cancer in a father or brother also have an increased risk of breast cancer. Altogether, less than 15% of women with breast cancer have a family member with the disease. This means that most (over 85%) women who get breast cancer do not have a family history of this disease [7]. A woman with cancer in one breast has a 3- to 4-fold increased risk of developing breast cancer in the other breast or in another part of the same breast [8]. Certain inherited DNA changes can increase the risk for developing cancer and are responsible for the cancers that run in families. For example, the breast cancer genes one and two (BRCA1 and BRCA2) are tumor suppressor genes. Mutations in these genes can be inherited from parents. When they are mutated, they no longer suppress abnormal growth and cancer is more likely to develop [9]. 

### 2.1. Estrogen as a Risk Factor

 The hormone estrogen works as a chemical messenger in the body. It is essential for normal sexual development and functioning of female organs important for childbearing like the ovaries, uterus, and breasts. Estrogen also helps regulate a woman's menstrual cycles. It is necessary for the normal development of the breast. It also helps maintain the heart and healthy bones. However, during each monthly menstrual cycle, a woman is exposed to increased estrogen levels, especially just before an egg is produced by her ovaries (ovulation). Also during pregnancy, women have prolonged exposure to high levels of estrogen. If a woman gives birth before 32 weeks or has an induced abortion, she will have an increased estrogen exposure without the protective effect of lobule differentiation. Estrogen can cause cancer in two ways. It acts as a “mitogen”; that is, it stimulates breast tissue to increase cell divisions (mitosis). This sometimes results in cancers due to errors in cell division (mutation). Secondly, certain metabolites of estrogen also act as carcinogens or genotoxins, by directly damaging DNA, thereby causing cancer cells to form [10]. Estrogen exposure can be in the form of environmental estrogens termed “xenoestrogens” which are naturally occurring like phytoestrogens in plants or synthetic chemicals that can act like human estrogen made by the ovary. Xenoestrogens can mimic the effect of human estrogen as they have a chemical structure that allows them to fit into the estrogen receptor the way a key fits into a lock.

The presence of estrogens can also activate hormones like relaxin to stimulate cell division. In fact, relaxin (RLX) has been shown to have a powerful effect on growth and differentiation of breast cancer (MCF-7) cells [14]. However, the effect of RLX is induced by estrogen probably by inducing RLX receptors as in myometrial cells [15]. Therefore, in general, it may be implicated in breast cancer risk because of its role in stimulating breast cell division, work during the critical periods of breast growth and development, effect on other hormones like relaxin that stimulate breast cell division, and support of the growth of estrogen-responsive tumors. Other studies have also shown that there is a positive relationship between endogenous hormone levels in postmenopausal women and risk of breast cancer [16]. In hormonal birth control mechanisms, there are two hormones involved, estrogen and progestin. Hormonal birth control mechanisms involve the oral contraceptives, minipill, Depo-Provera, and implants. These prevent pregnancy by releasing synthetic hormones to prevent the release of eggs from the ovaries (ovulation) and by thickening the cervical mucus, which helps block sperm from entering the uterus and by making it hard for an egg to attach and grow in the uterus. 

### 2.2. Researches on Other Risk Factors

 In the search for the actual cause of this deadly disease, many risk factors have been studied. Oral contraceptives use has undergone many discussions as a risk factor of breast cancer. A meta-analysis was performed of case control studies that addressed whether prior oral contraceptive use is associated with breast cancer. MEDLINE and PubMed databases and bibliography reviews were searched to identify related material published in or after 1980. Thirty-four studies were identified that met inclusion criteria. Two reviewers extracted data from original research articles or data provided by study authors. The DerSimonia-Laird method was used to compute pooled odds ratios (ORs) and confidence intervals (CIs). The Mantel-Haenszal test was then used to assess association between OC use and breast cancer. Results showed that the use of OCs was associated with an increased risk of premenopausal breast cancer in general with an OR (1.19) and 95% CI (1.09–1.29) and across various patterns used. It was associated with breast cancer risk in both parous (OR, 1.29; 95% CI, 1.20–1.40) and nulliparous women (OR, 1.24; 95% CI, 0.92–1.67) [17]. It was however not specific on whether the oral contraceptive investigated had estrogen, progesterone, or both. Other researchers have argued that estrogen level is increased in women receiving exogenous estrogens in form of OC or HRT [18]. Moreover, there is general agreement that the risk associated with OC and HRT depends on the duration of exposure, being lowest in women who never used OC or HRT [19]. 

Abortion and fertility have also been investigated as risk factors on breast cancer. In a research, modelling and forecasts based on abortion and other risk factors were done. They used the national cancer registration data for female breast cancer incidence in eight European countries: England and Wales, Scotland, Northern Ireland, the Irish Republic, Sweden, the Czech Republic, Finland and Denmark which were chosen because of their comprehensive data on abortion incidence. Relaxin has also been discovered to promote differentiation of breast cancer cells *in vitro*, more specifically, the MCF-7 breast adenocarcinoma cells. MCF-7 cells can be induced to progress in the differentiation pathway under the influence of relaxin (RLX), a peptide hormone that has been shown to have a powerful effect on growth and differentiation of epithelial and myoepithelial cells of the mouse mammary ducts *in vivo* [20]. Estrogen involvement has also been suggested. In fact, as shown for normal mammary gland, estrogens are needed to allow relaxin to produce its effect [14], probably by inducing relaxin receptors, as occurs in myo-metrial cells [15].

Association of metal exposure with breast cancer risk is a topic currently under discussions. An experiment was done to review the scientific evidence with respect to the *in vitro* and *in vivo* studies and epidemiological evidence for links between breast cancer and exposure to metals. It was found that there is growing evidence that environmental contaminants such as metals play a role in breast cancer [21]. Based on a relatively small number of studies, this literature review uncovered important deficiencies and gaps in the current literature that assesses the link of the incidence of breast cancer to metal exposure.

Several studies suggest that selective estrogen-receptor modulators (SERMs) like tamoxifen and raloxifene may lower breast cancer risk in women with certain breast cancer risk factors. But so far, many women are reluctant to take these medicines because they are concerned about possible side effects. Newer studies are looking at whether aromatase inhibitors; and drugs such as anastrozole, letrozole, and exemestane can reduce the risk of developing breast cancer in postmenopausal women. These drugs are already being used as adjuvant hormone therapy to help prevent breast cancer recurrences, but none of them is approved for reducing breast cancer risk at this time. One of these drugs, exemestane, has recently been shown to lower the risk of invasive breast cancer by 65% in women at increased risk. Fenretinide, a retinoid (drugs related to vitamin A), is also being studied as a way to reduce the risk of breast cancer. In a small study, this drug reduced breast cancer risk as much as tamoxifen. Other drugs are also being studied to reduce the risk of breast cancer [1].

Studies continue to uncover lifestyle factors and habits that alter breast cancer risk. Ongoing studies are looking at the effect of exercise, weight gain or loss, and diet on breast cancer risk. Studies on the best use of genetic testing for BRCA1 and BRCA2 mutations continue at a rapid pace. Scientists are also exploring how common gene variations may affect breast cancer risk. Each gene variant has only a modest effect in risk (10 to 20%), but when taken together they may potentially have a large impact. Potential causes of breast cancer in the environment have also received more attention in recent years. While much of the science on this topic is still in its earliest stages, this is an area of active research [3].

## 3. Treatment of Breast Cancer

 Treatment of breast cancer can be classified into broad groups, based on how they work and when they are used. These include surgery, chemotherapy, radiation therapy, and hormone therapy. Surgery is when the breast tumor is removed as partial mastectomy/breast-conserving surgery and mastectomy. Partial mastectomy surgery only removes a part of the affected breast, but how much is removed depends on the size and location of the tumor and other factors whilst mastectomy surgery removes the entire breast. The whole breast tissue is removed, and sometimes along with other nearby tissues. This can be in the form of a simple mastectomy or skin-sparing mastectomy depending on whether there is need for immediate reconstruction of the breast.

Radiation therapy, as the name implies, is treatment with high energy rays or particles that destroy cancer cells. This is also used to treat cancer that has spread to other areas, for example, to the bones or brain. It can be administered in two ways, external beam radiation and internal radiation. External beam radiation is when the radiation is focused from a machine outside the body on the area affected by the cancer. This procedure is more like getting an X-ray, but here the radiation is more intense. Brachytherapy, also called internal radiation, is when instead of aiming radiation beams from outside the body, radioactive seeds or pellets are placed directly into the breast tissue next to the cancer. Its administration is limited by tumor size, location of tumor, and other factors relating to the patient's medical condition. Systematic therapy refers to drugs which can be given by mouth or directly into the bloodstream to reach cancer cells anywhere in the body. chemotherapy, hormone therapy, and targeted therapy are examples.

Chemotherapy is treatment with cancer-killing drugs that can be given intravenously (injected into a vein) or by mouth. It is given in cycles, with each period of treatment followed by a recovery period. Treatment usually lasts for several months when chemotreatment is given to patients with no evidence of cancer after surgery. This is known as adjuvant therapy. When the treatment is given before surgery, chemotherapy is called neoadjuvant therapy. Hormone therapy hormonal therapy is often used as an adjuvant therapy to help reduce the risk of the cancer coming back after surgery although it can also be used as neoadjuvant treatment as well. This is when several approaches to blocking the effect of estrogen or lowering estrogen levels are used to treat hormone receptor-positive breast cancers. However, hormonal therapy does not help patients whose tumors are both estrogen receptor (er) negative and progestin receptor (PR) negative.

## 4. Models Done on Tumor Growth

 Several mathematical techniques have been applied in the study of breast cancer [11, 22–24]. Delay differential equations were used to model the interaction of breast cancer cells with the immune system. A developed model with delay differential equations modelling breast cancer accounted for different cell cycles and included terms to evaluate drug treatments, but ignored quiescent tumor cells [11]. Another related model included quiescent cells but ignored immune response and drug treatments in which there was consideration of the interconnected growth patterns of both proliferating and quiescent cells [22]. In a bid to improve the researches done by [11, 22], an integrated model in form of delay differential equations was developed accounting for quiescent cells, immune cells and included drug intervention terms. They included additional terms to account for the impact of Paclitaxel on the quiescent cells [25].

In one of the studies on the relationship between Body Mass Index (BMI), menopausal status, estrogen replacement therapy (ERT), and breast cancer risk, a mathematical model was developed and results showed that estrogen levels are responsible for the relationship between BMI, ERT, menopausal status, and breast cancer risk [23]. Statistical analysis and stochastic modelling have also been applied to investigate breast cancer and tumor growth [26]. They dealt with aspects of probability and statistics applied to breast cancer research. From *in vitro* experiments, breast cancer cells, the MCF-7 cells' behaviour in different types of substrates was noted. More specifically, it is how the stiffness of the different substrates affects the cell that is of most interest. The effect on aggregate counts and morphological parameters of the cells by surrounding (simulated) tissue's stiffness was analysed using methods from linear Mixed Models theory. The analysis indicated that certain parameters are significantly different for different tissue stiffness. Stochastic modelling related to initial tumor growth was studied and certain types of randomness were introduced in it. They numerically investigated how the model responds to stochastic behaviour of the parameters defining mutation characteristics. The model for tumor growth was rather stable with respect to small random perturbations. For the case of significant parameter randomness, the average number of cells (normal and mutant) at a time *T* was highly dependent on the expected value of the stochastic process representing the corresponding parameter value. This suggested a stable state for *in vitro* experiments and since *in vivo* experiments are known to be unstable, the presence of risk factors had aided in tumor behaviour.

A mathematical model of immune response to tumor invasion was also developed using competition models. Tumor cells population, CD8^+^T cell population, and Natural Killer cell population competed in a way almost similar to that suggested by Lotka-Volterra's competition models [24]. This carries a fundamental aspect on the interaction between immune cells and tumor cells. The presence of tumor cells stimulates the immune response, represented by the positive nonlinear growth term for the immune cells. This type of response term is of the same form as the terms used in the respective model of [27].

Cell populations have also been known to compete for nutrients and natural cell requirements resulting in nutrient consumption models. Burton [28] first proposed that diffusion and nutrient consumption might be limiting solid tumor, and since then a large number of studies have described the spatiotemporal interactions between tumor cell populations and nutrients. Early models of nutrient-limited tumor growth calculated the nutrient concentration profiles as a function of tumor spheroid radius that was changing due to the rate of cell proliferation [29]. The later models have incorporated differing degrees of complexity for cell movement. Tumor cell proliferation and death are considered to be dependent on only one generic nutrient (most often oxygen). However, some consider the effect of several nutrients and pH on the cell population [30].

The Gail model is also one of the widely used models and established models for predicting breast cancer risk in women. It was developed from a nested case control study conducted on a cohort of white women who were receiving regular screening mammograms in order to calculate multivariate relative risks of breast cancer based on age at menarche, age at first live birth, number of first-degree relatives (mother and sisters) with breast cancer, number of breast biopsies, and whether or not a typical hyperplasia was present on any biopsy specimen [31]. However, this widely used model does not predict breast cancer risk in young women generally and should not be used for that purpose [32]. It also underestimates genetically inherited breast cancer because it does not take into account paternal history. The model was also not intended to predict risk in women under age 40, nor in African American women of all ages [33].

Cell-DEVS, an extension of the DEVS formalism, has been used to model tumor-immune systems that involve growing tumors interacting with immune cells [34]. This has an advantage in that it facilitates the formal specification and reuse of cellular models. A Cell-DEVS model was implemented and tested using the CD++ toolkit and simulation results indicated that the model captured the intended qualitative aspects of tumor growth and immune system response [35]. Simulation-based parameter estimation offers a powerful means of estimating parameters in complex stochastic models. The use of simulation for computing the maximum likelihood estimator in the natural history of breast cancer was discussed. From the analysis, simulation provided a straight forward means of computing such estimators for models of substantial complexity [36].

A commonly proposed model for tumor growth assumes that the rate of growth is proportional to the number of malignant cells [37]. But currently, the hardest challenge in modelling tumor growth and treatment is estimating parameters in models that are mathematically simple and broadly applicable [38]. Most of the risk factors have shown an association with estrogen as emphasised so we seek to develop Lotka-Volterra's competition model of the tumor cells and the immune response in order to assess the impact of estrogen on the dynamics of breast cancer tumor.

## 5. The Estrogen-Free Model

 Based on many previous useful models done on tumor growth we here consider a model which subdivides the total population *N*(*t*) of cells of the breast tissue at any given time *t* into three groups which include normal or host cells, tumor cells and immune cells classes. The normal cells class, denoted by *H*(*t*) is in form of epithelial cells that make up the breast tissue. The cells differentiate and die normally as they have unaltered DNA which controls all cell actions. We assumed that the normal and tumor cells compete for space and resources in a small volume and therefore assumed a competition model used by Gatenby [39]. The normal cells grow exponentially at a *per capita* growth rate of *α*_1_ as a result of DNA initiation [39]. *β*_1_ is the depletion rate resulting from competition for resources such as nutrients and oxygen or the accumulation of substances released from cell metabolism within themselves. 

Tumor cells, denoted by *T*(*t*) at any time *t*, represent a class of breast cancer cells with damaged DNA. There are about 51 breast cancer cell lines which mirror the 145 primary breast tumors [40]. These can be classified into 2 major branches, the luminal, which has estrogen receptors (ESR1 positive), and basal-like, without estrogen receptors (ESR1 negative). We then assume a homogeneous luminal type of cancer cells in form of MCF-7, MDAMB361, BT474, T47D, and ZR75 cell lines. Several tumor growth laws have been proposed which include an exponential growth, Gompertz growth and logistic growth. We assume the presence of a small tumor mass, that is, a tumor size that is close to zero relative to carrying capacity, and therefore the choice of growth law does not significantly affect the qualitative behaviour of the model since they only differ for large tumor sizes. We therefore assume an exponential growth of tumor cells with *per capita* rate of *α*_2_ which results from the damaged DNA. Analogously *β*_2_ is a factor restricting their growth competition for space and food within themselves. The normal cells *H*(*t*) and tumor cells *T*(*t*) also compete for space and natural cell requirements like oxygen as they are supplied by the blood vessels. We assume cancer cells have uncontrolled cycle than the normal cells due to changed DNA which makes them fail to regulate a cell cycle [12] and thus their interaction with normal cells results in an inhibitory effect on normal cells at rate *δ*_1_ [41].

The model includes an immune cells class, *I*(*t*), in form of Natural Killer (NK) cells and CD8^+^ T cells. Their growth may be stimulated by the presence of the tumor and they can destroy tumor cells through a kinetics process. We also assume that the presence of a detectable tumor in a system does not necessarily imply that the tumor has completely escaped active immunosurveillance. Although a tumor is immunogenic, it is possible that the immune response may not be sufficient on its own to completely combat the rapid growth of the tumor cell population and the eventual development into a tumor.

The population of immune cells is considered to be outside of the system and we assume a background level of NK cells, even in the absence of tumor with CD8^+^ T cells only present as a result of activation. It is therefore reasonable to assume a constant source, *s*, of the immune cells from the thymus gland [27]. Furthermore, in the absence of any tumor, the cells will die off naturally at a *per capita* rate of *μ*. The presence of tumor cells stimulates the immune response resulting in growth of immune cells. This is represented by a positive nonlinear growth term for immune cells which as a function of *T*(*t*), is positive, increasing and concave with the form *ρI*(*t*)*T*(*t*)/(*ω* + *T*(*t*)), where *ρ* is the immune response rate and *ω* is the immune threshold rate, which is inversely proportional to the steepness of the immune response curve. This type of response term is of the same form as the terms used in respective models of [13, 27]. Thus immune cell proliferation is controlled and will never result in immune crowding which might in turn be detected as a threat. Furthermore, the reaction of immune cells and tumor cells can result in either the death of tumor cells at a rate *γ*_2_ or the inactivation of the immune cells, with *γ*_3_ as the interaction coefficient.

After considering all these aspects, we present the following system of Lotka-Volterra type of differential equations to determine the dynamics of breast cancer cells:

(1) $$\begin{array}{c} \frac{dH}{dt}=H\left(\alpha_{1}-\beta_{1}H-\delta_{1}T\right),\\ \frac{dT}{dt}=T\left(\alpha_{2}-\beta_{2}T\right)-\gamma_{2}IT,\\ \frac{dI}{dt}=s+\frac{\rho IT}{\omega +T}-\gamma_{3}IT-\mu I. \end{array}$$

Initial values of variables are *H*(0) = 1, *T*(0) = 10^−5^ and *I*(0) = *s*/*μ* = 1.379310345 adopted from [11, 13].

### 5.1. Equilibrium Points and Positivity of Solutions

 An equilibrium point is a stable condition that does not change over time, or in which change in one direction is continually balanced by change in another. The variables *H*, *T*, and *I* represent subpopulations of breast cells and therefore, should be positive or zero for all *t* ≥ 0. One can easily show that all the variables are greater than or equal to zero. If this condition is not met, the model should be discarded as it violates a basic aspect of scientific reality. The steady states occur where the ordinary differential equations are simultaneously zero, that is, where

(2) $$\begin{array}{c} \frac{dH}{dt}=\frac{dT}{dt}=\frac{dI}{dt}=0. \end{array}$$

The model system admits four steady states in which there are two dead equilibria, one tumor-free equilibrium points and one coexisting equilibrium point. 

#### 5.1.1. Tumor-Free Equilibrium-*ξ*_*t*_

 The first equilibrium point as the tumor-free equilibrium as this is when only tumor cell population has been forced to extinction as a result of the competition with normal and immune cells. This is given by

(3) $$\begin{array}{c} \xi_{t}=\left(H^{*},T^{*},I^{*}\right)=\left(\frac{\alpha_{1}}{\beta_{1}},0,\frac{s}{\mu }\right). \end{array}$$

We define a feasible region as a set of nonnegative and real solutions of our variables (*H*, *T*, *I*) since cell populations are nonnegative and real. The equilibrium state *ξ*_*t*_ exists since *α*_1_ > 0, *β*_1_ > 0, *μ* > 0, and *s* > 0, we have all solutions in the neighbourhood of *ξ*_*t*_ as positive and real and hence in the feasible region. 

#### 5.1.2. Type 1 Dead Equilibrium-*ξ*_*d*_^1^

 The dead equilibrium point is when normal cells only have died off leaving the tumor cells surviving. We classify this as a “dead” in the sense that there is no recovery of damaged normal cells since they have been forced to extinction. This is given by

(4) ξd1=(H∗,T∗,I∗)=(0,α2−γ2I∗β2,sμ−ρT∗/(ω+T∗)+γ3T∗),

where *ξ*_*d*_^1^ represents the type 1 dead equilibrium value of the normal cells, tumor cells, and immune cells, respectively.

The tumor cell population will increase with a decrease in tumor cell death rate, *β*_2_, and an increase in tumor growth rate, *α*_2_. An increase in immune cells also reduces tumor cell population as a result of predation on tumor cells by immune cells. We know that *β*_2_ > 0. So we need *α*_2_ ≥ *γ*_2_ I* which implies I* ≤ *α*_2_/*γ*_2_ so that T* can be in the feasible region. That is, the net growth rate of tumor cells must be more than or equal to immune cells at any time *t* in order for the competition to drive normal cells to extinction.

The immune cells are inversely proportional to tumor dynamics such that an increase in tumor dynamics reduces immune cells as more immune cells are deactivated by tumor cells. This exists when

(5) $$\begin{array}{c} \mu -\frac{\rho T^{*}}{\omega +T^{*}}+\gamma_{3}T^{*}>0, \end{array}$$

which when expanded will give

(6) $$\begin{array}{c} \gamma_{3}T^{*2}+\left(\mu +\omega \gamma_{3}-\rho \right)T^{*}+\mu \omega >0. \end{array}$$

By letting *u*_1_ = *γ*_3_, *u*_2_ = *μ* + *ωγ*_3_ − *ρ* and *u*_3_ = *μω*, we get

(7) $$\begin{array}{c} T^{*}=\frac{-u_{2}+\sqrt{u_{2}^{2}-4u_{1}u_{3}}}{2u_{1}}. \end{array}$$

We know that *u*_1_ > 0 and *u*_3_ > 0 and thus we need *u*_2_ < 0, that is, *μ* + *ωγ*_3_ < *ρ*. This implies that the immune response rate should be greater than the rate at which they are reduced. We also have *u*_2_^2^ − 4*u*_1_ *u*_3_ > 0 for T* to be real, that is, (*μ* + *ωγ*_3_ − *ρ*)^2^ > 4*γ*_3_ *ωμ* for solutions of our system around the type 1 dead equilibrium to be real and nonnegative. This implies that the difference in the rates of immune cell initiation and reduction should be greater than the rate at which they are lost. Also

(8) $$\begin{array}{c} \sqrt{u_{2}^{2}-4u_{1}u_{3}}\geq u_{2}\Rightarrow 4\mu \omega \gamma_{3}\leq 0, \end{array}$$

which means one or more of the parameters *μ*, *ω*, *γ*_3_ is zero. This explains that *ξ*_*d*_^1^ only exists when there are totally no immune dynamics which is a rare scenario, hence it is very rare to reach to such an equilibrium point unless someone is dead. 

#### 5.1.3. Type 2 Dead Equilibrium-*ξ*_*d*_^2^

 Type 2 dead equilibrium exists when both normal cells and tumor cell population have died off, given by

(9) $$\begin{array}{c} \xi_{d}^{2}=\left(H^{*},T^{*},I^{*}\right)=\left(0,0,\frac{s}{\mu }\right), \end{array}$$

where *ξ*_*d*_^2^ represents the type 2 dead equilibrium values for the normal cells, tumor cells and immune cells, respectively. Since *s* > 0 and *μ* > 0 it implies that all the solutions around the dead equilibrium of type 2, *ξ*_*d*_^2^ are in the feasible region. This state is feasible but however no fixed tissue is present which can be as a result of whole breast tissue removal maybe by a mastectomy surgery or death.

#### 5.1.4. Coexisting Equilibrium-*ξ*_*c*_

 The coexisting equilibrium point *ξ*_*c*_ is a state in which all cell populations have survived the competition and they coexist and is given by

(10) $$\begin{array}{c} \xi_{c}=\left(H^{*},T^{*},I^{*}\right)=\left(\frac{\alpha_{1}}{\beta_{1}}-\frac{\delta_{1}\left(\alpha_{2}-\gamma_{2}I^{*}\right)}{\beta_{1}\beta_{2}},\frac{\alpha_{2}-\gamma_{2}I^{*}}{\beta_{2}},\frac{s}{\mu -\rho T^{*}/\left(\omega +T^{*}\right)+\gamma_{3}T^{*}}\right), \end{array}$$

where *ξ*_*c*_ represent the coexisting equilibrium values of the normal cells, tumor cells and immune cells, respectively.

This exists when *β*_1_, *β*_2_ > 0 and

(11) $$\begin{array}{c} \alpha_{1}-\frac{\delta_{1}\left(\alpha_{2}-\gamma_{2}I^{*}\right)}{\beta_{2}}\geq 0,\\ \Rightarrow \frac{\alpha_{2}\delta_{1}-\alpha_{1}\beta_{2}}{\gamma_{2}\delta_{1}}\leq I^{*}. \end{array}$$

This implies that the combination of the net growth of tumor cells as a result of competition due to normal cells must always be less than the equilibrium value of the immune cells for the cells to coexist. I* > 0 when *α*_2_ *δ*_1_ ≥ *α*_1_ *β*_2_ which implies *α*_2_/*β*_2_ ≥ *α*_1_/*δ*_1_  . That is, the net growth of tumor cells must be greater than that of normal cells for a nonnegative solution to exist at *ξ*_*c*_. The equilibrium values for the tumor cells and immune cells are given as the same as the ones at the type 1 dead equilibrium. 

### 5.2. Stability Analysis of Equilibria

 We analyse the equilibrium points in terms of their stability by means of eigenvalues. We apply the Hartman Grobman Theorem which states that in the neighbourhood of a hyperbolic equilibrium point, a nonlinear dynamical system is topologically equivalent to its linearisation. 

#### 5.2.1. Local Stability of the Tumor-Free Equilibrium Point

 We now evaluate the stability of the tumor-free equilibrium point, that is at *ξ*_*t*_ in which the Jacobian is given by

(12) $$\begin{array}{c} J_{\xi_{t}}=\;\;\left(\begin{array}{ccc} -\alpha_{1} & -\frac{\alpha_{1}\delta_{1}}{\beta_{1}} & 0\\ 0 & \alpha_{2}-\frac{\gamma_{2}s}{\mu } & 0\\ 0 & \frac{s}{\mu }\left(\frac{\rho }{\omega }-\gamma_{3}\right) & -\mu \end{array}\right). \end{array}$$

Therefore the system gives three eigenvalues (*λ*_*i*_) which are, *λ*_1_ = −*α*_1_, *λ*_2_ = *α*_2_ − *γ*_2_ *s*/*μ*, and *λ*_3_ = −*μ*. Since *λ*_1_, *λ*_3_ < 0, we have the tumor-free equilibrium point being stable as long as *α*_2_ < *sγ*_2_/*μ*. This implies that the system is stable at tumor-free if and only if the resistance coefficient *sγ*_2_/*μ* is greater than the *per capita* growth rate of the tumor cells, *α*_2_. This measures how the immune system competes with the tumor cells and since we assumed that the immune cells are capable of destroying cancer cells at some rate, we have *λ*_2_ being negative and therefore *ξ*_*t*_ is always a stable equilibrium point. 

#### 5.2.2. Local Stability of Type 1 Dead Equilibrium

 Evaluating the Jacobian at the *ξ*_*d*_^1^ gives the first eigenvalue as

(13) $$\begin{array}{c} \Rightarrow \lambda_{1}=\frac{\alpha_{1}\beta_{2}-\alpha_{2}\delta_{1}+\delta_{1}\gamma_{2}I^{*}}{\beta_{2}}. \end{array}$$

We know from Section 5.1.4 that *α*_1_ *β*_2_ − *α*_2_ *δ*_1_ + *δ*_1_ *γ*_2_ I* ≥ 0, thus *λ*_1_ is a nonnegative eigenvalue and thus the type 1 dead equilibrium is always unstable. This is in fact the case suggested by De Pillis and Radunskaya [13] that the dead equilibria are always unstable in host dynamics. This implies that once interactions among these cells drives them to the death of normal cells, there is no recovery and no form of intervention or parameter adjustment that will stabilise it. That is, once normal cells' DNA is damaged, the cell can never recover. 

#### 5.2.3. Local Stability of Type 2 Dead Equilibrium

 Evaluating the Jacobian at the point *ξ*_*d*_^2^ gives

(14) $$\begin{array}{c} J_{\xi_{d}^{2}}=\left(\begin{array}{ccc} \alpha_{1} & 0 & 0\\ 0 & \alpha_{2}-\frac{\gamma_{2}s}{\mu } & 0\\ 0 & \frac{s}{\mu }\left(\frac{\rho }{\omega }-\gamma_{3}\right) & -\mu \end{array}\right). \end{array}$$

The system has three eigenvalues (*λ*_*i*_) which are *λ*_1_ = *α*_1_, *λ*_2_ = *α*_2_ − *γ*_2_ *s*/*μ*, and *λ*_3_ = −*μ* and since *α*_1_ > 0 and −*μ* < 0, this implies that whatever value of *λ*_2_, the type 2 dead equilibrium is a saddle point which is always unstable.

#### 5.2.4. Local Stability of the Coexisting Equilibrium Point

 We would want to analyse how the system behaves around the coexisting equilibrium point, *ξ*_*c*_. For simplicity, we introduce parameters *f*(*h*), *f*(*t*), *f*(*i*) where,

(15) f(t)=α2−γ2I∗β2,f(h)=α1β1−δ1(α2−γ2I∗)β1β2,f(i)=sμ−ρT∗/(ω+T∗)+γ3T∗.

We need *f*(*h*) ≥ 0, *f*(*t*) ≥ 0 and *f*(*i*) ≥ 0, for feasibility of solutions, and therefore these parameters are nonnegative as shown in the previous sections. Thus computing the Jacobian matrix at this point gives

(16) Jξc=(α1−2β1f(h)−δ1f(t)−δ1f(h)00α2−2β2f(t)−γ2f(m)−γ2f(t)0−ρωf(i)(f(t)+ω)2−f(i)γ3−μ+ρf(t)ω+f(t)−γ3f(t)).  

This results in one of the eigenvalues

(17) $$\begin{array}{c} \lambda_{1}=\alpha_{1}-2f\left(h\right)\beta_{1}-f\left(t\right)\delta_{1}. \end{array}$$

Substituting for *f*(*t*) and *f*(*h*), then solve we have

(18) $$\begin{array}{c} \lambda_{1}=-\alpha_{1}+\delta_{1}\left(\frac{\alpha_{2}-\gamma_{2}I^{*}}{\beta_{2}}\right). \end{array}$$

However, since H* exist at *ξ*_*c*_ when

(19) $$\begin{array}{c} \alpha_{1}-\frac{\delta_{1}\left(\alpha_{2}-\gamma_{2}I^{*}\right)}{\beta_{2}}\geq 0, \end{array}$$

this implies that *λ*_1_ is negative and thus the stability of the system can be determined by the state of eigenvalues *λ*_2_ and *λ*_3_. These are obtained from the remaining 2 × 2 matrix below:

(20) τ=(α2−2β2f(t)−γ2f(i)−γ2f(t)−ρωf(i)(f(t)+ω)2−f(i)γ3−μ+ρf(t)ω+f(t)−γ3f(t)).

For the system to be stable, we need the trace to be negative and the determinant to be positive. The trace  (*τ*) can be written as

Trace (*τ*) = −*α*_2_ + 2*γ*_2_ I* − *γ*_2_ *f*(*i*) − *μ* + *ρf*(*t*)/(*ω* + *f*(*t*)) − *γ*_3_ *f*(*t*).

For stability, we need trace *τ* < 0,

(21) $$\begin{array}{c} \Rightarrow 2\gamma_{2}I^{*}-\gamma_{3}f\left(t\right)+\frac{\rho f\left(t\right)}{\omega +f\left(t\right)}-\mu <\alpha_{2}+\gamma_{2}f\left(i\right). \end{array}$$

That is, for us to have a stable system, tumor cell dynamics should be less than that of immune cell population. Also we need the determinant (Δ) of the 2 × 2 matrix to be positive for the system to be stable. The determinant Δ for the system is also given by

(22) Δ=f(i)γ2(f(t))2(μ−ρ)+2f(t)μω+μω2−γ2(f(t)+ω)f(t)(μ−ρ)+μω+f(t)(f(t)+ω)γ3+2f(t)β2(f(t)+ω)(f(t)(μ−ρ))+μω+f(t)γ3(f(t)+ω).

For Δ > 0

(23) f(i)γ2(f(t))2(μ−ρ)+2f(t)μω  +μω2+μω+f(t)γ3(f(t)+ω)  >γ2(f(t)+ω)f(t)(μ−ρ).

We know that *f*(*t*) is a function of I* and *f*(*i*) is a function of T*, therefore we generally have the growth of immune cells being greater than that of tumor cells for us to have a stable system. 

#### 5.2.5. Global Stability of Equilibria

 To establish the global asymptotic stability of the equilibrium points, we adopt the method of Castilo-Chavez [42]. We rewrite system (1) as

(24) $$\begin{array}{c} \frac{dX}{dt}=F\left(X,Z\right),\\ \frac{dZ}{dt}=G\left(X,Z\right), \end{array}$$

where *G*(*X*, 0) = 0, *X* ∈ *ℜ* ^2^ denotes the undamaged cell compartments, (*H*(*t*) and *I*(*t*)) and *Z* ∈ *ℜ* ^1^ is comprised of the damaged cell compartment, *T*(*t*).

The conditions below must be satisfied to guarantee global stability.

 
*H*1 : For *dX*/*dt* = *F*(*X*, 0), X* is globally asymptotically stable.
 
*H*2: *G*(*X*, *Z*) = *AZ* − G*(*X*, *Z*), *G*(*X*, *Z*) ≥ 0 for (*X*, *Z*) ∈ *Ω* where *A* = *D*_*Z*_ *G*(X*, 0) is an *M*-matrix (with off diagonal elements as nonnegative) and *Ω* is the region where the model makes biological sense.

In our case,

(25) $$\begin{array}{c} F\left(X,0\right)=\left(\begin{array}{c} \alpha_{1}H-\beta_{1}H^{2}\\ \;s-\mu I \end{array}\right) \end{array}$$

and *A* is a 1 × 1 matrix given by

(26) $$\begin{array}{c} A=D_{Z}G\left(X^{*},0\right)=\alpha_{2}-2\beta_{2}T^{*}-\gamma_{2}I^{*},\;\;\\ G^{*}\left(X,Z\right)=-\beta_{2}T^{*}. \end{array}$$

We therefore conclude that the tumor-free equilibrium, *ξ*_*t*_ is the only state that is globally asymptotically stable since G*(*X*, *Z*) ≥ 0. All the other equilibrium states are globally unstable since G*(*X*, *Z*) < 0.

Hence, the system can only be stable when the immune system can efficiently compete with the cancer cells, that is, the efficiency in CD8+ activation and NK cell supply from the thymus. As shown by both equilibria, immune resistance to tumor growth is the only factor that determines stability of the system. The general necessary condition for stability of our system is that the growth rate of immune cells *α*_2_ must be greater than the immune cell resistance coefficient *sγ*_2_/*μ*. The global stability of the system is only dependant on the natural exponential death of tumor cells. That is, as the number of tumor cells dies naturally, the system approaches a stable state.

## 6. Model with Estrogen

 We introduce another class of estrogen, *E*(*t*), in the form of 17-*β* estradiol to the dynamics of breast cancer cells. Over and above the estrogen produced by the ovaries, there is more estrogen introduced into the system as part of some oral contraceptives, in hormone replacement therapy or in estrogen replacement therapy. The assumption here is that as women take hormonal birth control methods they increase a constant level of the estrogen hormonal level. We therefore assume a constant source, *π* of 17-*β* estradiol, the primary biologically most active estrogen which is all the estrogen in the system at any given time.

Human breast cells, the epithelial cells, contain estrogen receptors termed estrogen receptor-1 (ER-*α*) and estrogen receptor-2 (ER-*β*). These are intracellular receptors, which when activated by ligand binding, translocate to the nucleus and act as transcription factors by binding to DNA in the promoter regions of target genes. Both ER-*α* and ER-*β* bind 17-*β* estradiol in the nucleus of the cell with similar affinity (0.1–1 nM) and act as transcription factors to regulate gene expression. This will lead to gene transactivation which may also result from tethering of estrogen receptors to nuclear transcription factors such as NFYB and SPI [43]. It is also consistent to assume that the estrogen modulation of the inflammatory response is a contributing factor in estrogen-stimulated growth of breast tumor [43] which also has an effect on the host innate immune response. This can however result in damage to DNA primary structure of the double helix as a result of estrogen oxidation products, the 2-OH and 4-OH catechol estrogens, and how it stimulates cell proliferation and gene expression via the ER. Therefore, normal cell population, *H*(*t*) will be reduced as some of the normal cells are being converted into tumor cells by a factor *σ*_1_ *HE*, where *σ*_1_ is the rate of tumor formation as a result of DNA damage by estrogen. Damaged normal cells will now form the class of tumor cells and therefore tumor cell population will also increase at a rate *σ*_2_ resulting in a growth factor of *σ*_2_ *HE* on tumor cell population. Here *σ*_2_ < *σ*_1_ since some of the damaged cells can be destroyed as a result of antitumor immunity from Natural Killer cells.

Estrogen is oxidised to catechol estrogens by recombinant phase 1 enzymes (CYP1A1 and CYP1B1) which also die naturally at a rate *θ* represented by the death factor *θE*. The molecule 17-*β* estradiol stimulates growth in estrogen-responsive breast cancer cells. As shown by [44] in a series of experiments, ER-positive cells can stimulate surrounding benign cells to proliferate through similar paracrine effects involving stromal-epithelial cell interactions. ER-positive breast cancer cells are themselves stimulated to grow by estrogen through autocrine effects, and they are Ki67 positive [45]. We therefore introduce a growth factor *α*_3_ *T* of tumor cells where *α*_3_ is the *per capita* growth of *T*(*t*) cells which is greater than *α*_2_, the growth factor from the estrogen-free model. *α*_3_ is greater than *α*_2_ as a result of combined natural growth rate plus growth due to autocrine effects.

The presence of estrogen has also been shown to reduce immune cell proliferation. A process known as ovariectomy which involves removal of one or both ovaries upregulates *T* cell Tumor Necrosis Factor (TNF) production by increasing the number of TNF producing *T* cells without altering the amount of TNF produced by each *T* cell [46]. We therefore assume that if estrogen deficiency increases immune cell proliferation and lifespan, then its presence will inhibit immune cell proliferation. We can therefore represent this by a decay factor

(27) $$\begin{array}{c} \frac{\sigma_{3}IE}{\upsilon +E} \end{array}$$

on immune cells with *σ*_3_ as the rate of immune suppression due to estrogen presence and *υ* is the estrogen threshold rate. Incorporating these effects of estrogen on system (1) will result in the following system of equations:

(28) dHdt=H(α1−β1H−δ1T)−σ1HE,dTdt=T(α3−β2T)−γ2IT+σ2HE,dIdt=s+ρITω+T−γ3IT−μI−σ3IEυ+E,dEdt=π−θE,

where *H*(0) = 1, *T*(0) = 10, *I*(0) = 1.379310345, and *E*(0) = 2.

### 6.1. Equilibrium Points and Positivity of Solutions

 The model system admits three steady states which are the dead equilibrium, tumor-free equilibrium, and coexisting equilibrium points.

#### 6.1.1. Tumor-Free Equilibrium *ψ*_*t*_

 The tumor-free equilibrium is when only the tumor cell population has died due to the competition with the other cells. This is given by

(29) ψt=(H•,T•,I•,E•)=(α1−σ1E•β1,0,s(E•+υ)μ(E•+υ)+σ3E•,πθ),

where *H* ^•^, *T* ^•^, *I* ^•^, *E* ^•^ represent the tumor free equilibrium values for the normal cells, tumor cells, immune cells, and the estrogen hormone, respectively. We have *I* ^•^ > 0 and *E* ^•^ > 0 since all parameters *s*, *υ*, *μ*,*σ*_3_, *θ*, *π*, *σ*_1_, *α*_1_, and *β*_1_ are positive. *I* ^•^ now depends on estrogen suppression unlike in the estrogen-free model, where it only depends on natural dynamics.

*H* ^•^ will be nonnegative at *ψ*_*t*_ when (*α*_1_ − *σ*_1_ *E* ^•^)/*β*_1_ ≥ 0,

(30) $$\begin{array}{c} \Rightarrow E^{•}\leq \frac{\alpha_{1}}{\sigma_{1}}. \end{array}$$

This implies that estrogen cells at any given time *t* should be less than the growth coefficient of normal cells. We also noted earlier on that *E* ^•^ is nonnegative. Therefore, the existence of a tumor-free equilibrium in this case depends on the estrogen levels and (30) whilst on the estrogen-free model it depends on the natural dynamics only. 

#### 6.1.2. Dead Equilibrium *ψ*_*d*_

 An equilibrium point is referred to as dead if the host cell population is zero. There are two dead equilibria where the first one is as a result of breast tissue removal characterised with both normal cells and tumor cell population having died off. This is feasible as the competition has led to exclusion of both normal and tumor cells but however not of importance since it does not give us anything to analyse the effects of estrogen on the dynamics of breast cancer. The second dead equilibrium is given by

(31) $$\begin{array}{c} \psi_{d}=\left(H^{•},T^{•},I^{•},E^{•}\right)=\left(0,\frac{\gamma_{2}I^{•}-\alpha_{3}}{\beta_{2}},\frac{s}{\mu +\delta_{3}E^{•}/\left(\nu +E^{•}\right)+\gamma_{3}T^{•}-\rho T^{•}/\left(\omega +T^{•}\right)},\frac{\pi }{\theta }\right), \end{array}$$

where (*H* ^•^, *T* ^•^, *I* ^•^, *E* ^•^) represents the equilibrium values of the normal cells, tumor cells, immune cells and estrogen levels, respectively. This dead equilibrium is a situation where the normal cells have been out competed by the tumor cells and as a result the whole breast tissue is a tumor. It exist when *I* ^•^ < *α*_3_/*γ*_2_ and *μ* + *δ*_3_ *E* ^•^/(*ν* + *E* ^•^) > (*ρT* ^•^/(*ω* + *T* ^•^) − *γ*_3_ *T* ^•^). Which implies the net growth of the tumor cells must be more than the immune cell value in order to have the tumor cells outgrowing the normal cells as the reactivation of the immune cells due to estrogen effects is greater than the reactivation of the immune cells due to tumor effect.

#### 6.1.3. Coexisting Equilibrium-*ψ*_*c*_

 The coexisting equilibrium state exists when all cell populations would have survived the competition. This is given by *ψ*_*c*_ = (*H* ^•^, *T* ^•^, *I* ^•^, *E* ^•^) where *H* ^•^, *T* ^•^, *I* ^•^, and *E* ^•^ represent the coexisting equilibrium values for the normal cells, tumor cells, immune cells and the estrogen hormone, respectively, and are given by,

(32) H•=α1−δ1T•−σ1E•β1,T•=12β1β2(−B+B2−4β1β2(−α1σ2E•+σ1σ2E•2)),I•=sμ−ρT•/(ω+T•)+γ3T•+σ3E•/(υ+E•),E•=πθ,

where *B* = −*α*_3_ *β*_1_ + *β*_1_ *γ*_2_ *I* ^•^ + *δ*_1_ *σ*_2_ *E* ^•^. Since *π* and *θ* are positive parameters, we have *E* ^•^ ≥ 0. We also need *α*_1_ ≥ *δ*_1_ *T* ^•^ + *σ*_1_ *E* ^•^ for *H* ^•^ to be feasible at this equilibrium state. That is, the rate of normal cell growth must be greater than the rate at which they are lost as a result of interactions with tumor and presence of more estrogen. The value of *T* ^•^ > 0 at the *ψ*_*c*_ when

(33) $$\begin{array}{c} E^{•}\left(\sigma_{1}\sigma_{2}E^{•}-\alpha_{1}\sigma_{2}\right)\geq 0. \end{array}$$

Therefore we have either *E* ^•^ = 0 resulting in estrogen-free model or *E* ^•^ ≥ *α*_1_/*σ*_1_  which implies that the estrogen levels must be greater than the net growth rate of normal cells for cells to coexist an opposite case with the tumor-free state equation (30).

*I* ^•^ exists at *ψ*_*c*_ when

(34) $$\begin{array}{c} \mu +\frac{\sigma_{3}E^{•}}{\upsilon +E^{•}}>\frac{\rho T^{•}}{\omega +T^{•}}-\gamma_{3}T^{•}. \end{array}$$

Therefore activation of immune response as a result of tumor presence should be lower than the rate at which they are lost due to estrogen effects plus natural death. 

### 6.2. Stability Analysis of Equilibria

 Linearising the system at different equilibrium values gives the following. 

#### 6.2.1. Local Stability of the Tumor-Free Equilibria

 We would want to check how the system at the tumor-free equilibrium point will now behave in terms of stability given the incorporated effects of estrogen. The system has four eigenvalues (*λ*_*i*_) which will determine the stability of the system, with the first two eigenvalues both negative and given as

(35) $$\begin{array}{c} \lambda_{1}=-\theta ,\;\;\lambda_{2}=-\frac{{\mu \left(\pi +\theta \upsilon \right)+\sigma }_{3}\pi }{\pi +\theta \upsilon }. \end{array}$$

The remaining eigenvalues are given by the characteristic equation:

(36) λ2−λ(α3+3σ1E•+γ2g(i)−α1)  +α1α3−2g(h)α3β1−α1α2g(i)  +2g(i)g(h)β1γ2−α3σ1πθ  +g(i)γ2σ1πθ+g(h)δ1σ2πθ=0,

where

(37) g(h)=α1−σ1E•β1,g(i)=s(E•+υ)μ(E•+υ)+σ3E•.

Since (*α*_3_ − *α*_1_ + 3*σ*_1_ *E* ^•^ + *γ*_2_ *g*(*i*)) is positive due to the fact that the rate of tumor growth is greater than that of normal cells, that is, *α*_2_ > *α*_1_, this implies −(*α*_3_ − *α*_1_ + 3*σ*_1_ *E* ^•^ + *γ*_2_ *g*(*i*)) is negative and by Routh Hurwitz criterion the system cannot be stable. Thus the tumor-free equilibrium point is always unstable implying the existence of estrogen has caused instability in the tumor free state. 

#### 6.2.2. Local Stability of the Coexisting Equilibrium Point

 We linearise the system of differential equations (28) at *ψ*_*c*_ = (*H* ^•^, *T* ^•^, *I* ^•^, *E* ^•^) = (*p*(*h*), *p*(*t*), *p*(*i*), *π*/*θ*), where from the previous section, *p*(*h*), *p*(*t*) and *p*(*i*) are nonnegative and real parameters. This results in the following eigenvalues with *λ*_1_ = −*θ* which is negative. The other eigenvalues are obtained from the following characteristic equation:

(38) λ3+λ2(α1+α3−2p(h)β1−2p(t)β2−p(i)γ2     −p(t)δ1−2p(t)2β2δ1−σ1E•−sI•)+⋯=0.

By Routh-Hurwitz criteria the system is stable only if

(39) α1+α3>2p(h)β1+2p(t)β2+p(i)γ2  +p(t)δ1+2p(t)2β2δ1+σ1E•+sI•

It is ideal when we have the growth of the tumor and normal cells being greater than their depreciation if they have to survive competition and coexist regardless of the interactions. Otherwise if the rate of growth of these normal and tumor cells is lower than the rate at which they die due to either interaction or naturally, this will lead to competitive exclusion and hence the dead equilibria. We therefore conclude that it is ideal to have

(40) α1+α3<2p(h)β1+2p(t)β2+p(i)γ2+p(t)δ1+2p(t)2β2δ1+σ1E•+sI•,

which implies a negative coefficient for *λ*_2_; hence the system is unstable if cells coexist. 

#### 6.2.3. Global Stability of Equilibria

 Global stability of the equilibrium points here is done using Castilo-Chavez method [42]. We rewrite system (1) as

(41) $$\begin{array}{c} \frac{dX}{dt}=F\left(X,Z\right),\\ \frac{dZ}{dt}=G\left(X,Z\right), \end{array}$$

where *G*(*X*, 0) = 0, *X* ∈ *ℜ* ^3^ denotes the undamaged cell compartments (*H*(*t*), *I*(*t*) and *E*(*t*)), and *Z* ∈ *ℜ* ^1^ is comprised of the damaged cell compartment; *T*(*t*).

The conditions below must be satisfied to guarantee global stability.

 H1: For *dX*/*dt* = *F*(*X*, 0), *X* ^•^ is globally stable.
 H2: *G*(*X*, *Z*) = *AZ* − *G* ^•^(*X*, *Z*), *G*(*X*, *Z*) ≥ 0 for (*X*, *Z*) ∈ *Ω*.

where *A* = *D*_*Z*_ *G*(*X* ^•^, 0) is an *M*-matrix (with off diagonal elements as nonnegative) and *Ω* is the region where the model makes biological sense. In our case,

(42) $$\begin{array}{c} F\left(X,0\right)=\left(\begin{array}{c} \alpha_{1}H-\beta_{1}H^{2}-\sigma_{1}HE\\ s-\mu I-\frac{\sigma_{3}IE}{\upsilon +E}\\ \pi -\theta E \end{array}\right), \end{array}$$

and *A* is a 1 × 1 matrix given *A* = *D*_*Z*_ *G*(*X* ^•^, 0) = *α*_2_ − 2*β*_2_ *T* ^•^ − *γ*_2_ *I* ^•^ and *G* ^•^(*X*, *Z*) = −(*β*_2_ *T* ^•^ + *σ*_2_ *H* ^•^ *E* ^•^).

The conditions H1 and H2 have not been satisfied. We therefore conclude that the tumor-free equilibrium, *ψ*_*t*_ is globally unstable since *G* ^•^(*X*, *Z*) < 0. The coexisting equilibrium point *ψ*_*c*_ likewise is globally unstable since *G* ^•^(*X*, *Z*) < 0 for all nonnegative values of coexisting equilibrium points. The global stability of the system now depends for the presence of estrogen levels

## 7. Numerical Simulations

 Matlab 6.5 version was used for all our simulations for both models using ODE45 solver. Simulations on this model give us a portrait of the general behaviour of breast cancer cells in the presence of normal cells and immune cells. We are also concerned on the parameters which are of importance in stabilising the model and the ranges in which the system is stable and unstable. Initial values of variables are *H*(0) = 1, *T*(0) = 10^−5^, and *I*(0) = *s*/*μ* = 1.379310345 adopted from [13]. All parameter values used for the numerical simulations are as shown in Table 1. The numerical solutions generally show that in the presence of excess estrogen, tumor cells grow as shown by Figure 1(a) while immune cells and normal cells decrease with normal cells being the most affected (Figure 1(b)).

## 8. Conclusions

 The general dynamics of breast cancer have been presented in form of a system of differential equations. Conditions of stability of the tumor-free equilibria were established. The system is only stable if and only if the immune resistance is greater than tumor growth rate. That is, the chance of an individual developing breast cancer depends on the ability of the immunity to combat tumor cells. We have also deduced that the presence of excess estrogen in the system makes it unstable. This implies that additional estrogen quantity introduced increases rate of tumor development hence the development of breast cancer. This is supported by Figure 2(a) which shows that the normal cells grow normally without excess estrogen levels (pi = 0). However, their growth is affected negatively in the presence of excess estrogen as they decrease with increase in estrogen amounts. The excess estrogen is however, a favorable condition to the tumor growth. When pi = 0 tumor cells can be controlled to minimum levels by the immune system but rises to uncontrollable levels as the estrogen amount increases bringing the instability as shown by Figure 2(b). This is so because excess estrogen increases the rate of tumor formation and also suppresses immune growth.  Figure 3(a) shows that immune levels are reduced with increase in estrogen levels hence weakening the immune system. Therefore the immune system will not be able to compete effectively with the cancer cells and thus will fail to control the disease. The estrogen-free model is always stable in the absence of any tumor but as we introduced estrogen, the system became unstable as shown on the global stability. Thus, the presence of excess estrogen will lead into a situation in which the disease is uncontrollable. No form of control measure or intervention can stabilise the system since it is always unstable in the presence of excess estrogen. Therefore, abnormal estrogen levels increase the chances of an individual developing breast cancer. This can also implies that the use of estrogen hormone as a birth control method has a negative impact since it can cause breast cancer. The global stability of the model system (28) shows that as estrogen levels approach zero, the tumor-free equilibrium becomes stable. This brings us to another aspect that increasing estrogen levels will increase the chance of an individual developing breast cancer.

Numerical simulations have also shown that tumor population increases as estrogen source rate increases in excess estrogen (Figure 2(b)). That is, as estrogen levels increase, the risk of developing breast cancer also increases. Normal and immune cells also decreased with an increase in estrogen levels. This implies that in the long run, the whole breast tissue will be infested with tumor cells in the presence of excess estrogen. We have also found out that any estrogen amount above normal has a negative impact on the dynamics of normal and immune cells. We therefore conclude that taking extra estrogen levels either as hormonal birth control or beauty enhancing practices will increase risk of breast cancer development. 

## 9. Discussion

 The results clearly show a negative relationship of estrogen amounts and tumor cell development. The development of tumor cells depends on the ability of the normal cells (immune system) to combat tumor cells in the absence of excess estrogen and on estrogen levels plus immune compatibility in case of excess estrogen levels. However, it must be noted that it may also depend on genetics of an individual like the ability of DNA to resist change in structure and amount of estrogen released during natural biological processes like menopause and premenopause stages. Exposure periods to radioactive material, for example, are other external factors which have not also been incorporated in the model which might result in a difference of the results.

## Figures and Tables

**Figure 1:** (a) Showing the general result tumor progression with excess estrogen. (b) Showing the general normal, immune, and estrogen levels in the presence of excess estrogen.

**Figure 2:** (a), (b) are graphs of numerical solutions showing the propagation of normal cells and tumor cells, respectively, with estrogen variations.

**Figure 3:** (a) The propagation of immune cells with estrogen variations. (b) The coexistence state of normal, tumor, and immune cells in the presence of excess estrogen.

**Table 1:** Model parameters and their interpretations.

Parameter	Symbol	Value	Units	Reference
*Per capita* growth rate of normal cells	α_1_	0.70	(day)^−1^	est
Per capita growth rate of tumor cells	α_2_	0.98	(day)^−1^	[11]
Natural death rate of normal cells	β_1_	0.30	(day)^−1^	est
Natural death rate of tumor cells	β_2_	0.40	(day)^−1^	[12]
Normal cell death rate due to competition	δ_1_	1.0	(day)^−1^	[12]
Tumor death rate due to immune response	γ_2_	0.9	(day)^−1^	[12]
Source rate of immune cells	*s*	0.4	(day)^−1^	[13]
Immune response rate	ρ	0.2	(day)^−1^	[13]
Immune threshold rate	ω	0.3	(day)^−1^	[13]
Natural death rate of immune cells	μ	0.29	(day)^−1^	[12]
